This article has been retracted.

# Prediction of Early Alzheimer Disease by Hippocampal Volume Changes under Machine Learning Algorithm

**DOI:** 10.1155/2022/3144035

**Published:** 2022-05-06

**Authors:** Qun Shang, Qi Zhang, Xiao Liu, Lingchen Zhu

**Affiliations:** Department of Radiology, Zibo Central Hospital, Zibo, 255000 Shandong, China

## Abstract

This research was aimed at discussing the application value of different machine learning algorithms in the prediction of early Alzheimer's disease (AD), which was based on hippocampal volume changes in magnetic resonance imaging (MRI). In the research, the 84 cases in American Alzheimer's disease neuroimaging initiative (ADNI) database were selected as the research data. Based on the scoring results of cognitive function, all cases were divided into three groups, including cognitive function normal (normal group), early mild cognitive impairment (e-MCI group), and later mild cognitive impairment (l-MCI group) groups. Each group included 28 cases. The features of hippocampal volume changes in MRI images of the patients in different groups were extracted. The samples of training set and test set were established. Besides, the established support vector machine (SVM), decision tree (DT), and random forest (RF) prediction models were used to predict e-MCI. Metalinear regression was utilized to analyze MRI feature data, and the predictive accuracy, sensitivity, and specificity of different models were calculated. The result showed that the volumes of hippocampal left CA1, left CA2-3, left CA4-DG, left presubiculum, left tail, right CA2-3, right CA4-DG, right presubiculum, and right tail in e-MCI group were all smaller than those in normal group (*P* < 0.01). The corresponding volume of hippocampal subregions in l-MCI group was remarkably reduced compared with that in normal group (*P* < 0.001). The volumes of regions left CA1, left CA2-3, left CA4-DG, right CA2-3, right CA4-DG, and right presubiculum were all positively correlated with logical memory test-delay recall (LMT-DR) score (*R*^2^ = 0.1702, 0.3779, 0.1607, 0.1620, 0.0426, and 0.1309; *P* < 0.001). The predictive accuracy of training set sample by DT, SVM, and RF was 86.67%, 93.33%, and 98.33%, respectively. Based on the changes in the volumes of left CA4-DG, right CA2-3, and right CA4-DG, the predictive accuracy of e-MCI and l-MCI by RF model was both higher than those by DT model (*P* < 0.01). Besides, the predictive accuracy, sensitivity, and specificity of e-MCI by RF model was all notably higher than those by DT model (*P* < 0.01). The above results demonstrated that the effective early AD prediction models were established by the volume changes in hippocampal subregions, which was based on RF in the research. The establishment of early AD prediction models offered certain reference basis to the diagnosis and treatment of AD patients.

## 1. Introduction

Alzheimer's disease (AD) is a common type of symptom among senile dementia. The clinical features of AD are progressive cognitive decline and behavior abnormality. The incidence of AD is positively correlated with age. The incidence of AD reaches about 13% among the population aged 65, and it is as high as 43% among the population aged 85 and above [1]. With the aggravation of current global population aging, the number of AD patients is growing obviously. In 2018, 50 million people suffered from AD all over the world. It is predicted that the number of AD patients will increase to 82 million by 2030 [2]. Mild cognitive impairment (MCI) is the early phase of the development of AD disease. Effective intervention measures for MCI patients can restore their cognitive state back to normal levels [3]. With the change in disease status, amyloid beta deposition affects hippocampal volumes to some extent. The changes in hippocampal volumes promote the early diagnosis of AD population [4]. With the continuous development of imaging and medical technologies in recent years, structural magnetic resonance imaging (MRI), positron emission tomography (PET), electroencephalogram (EEG), brain metabolic imaging, and cerebrospinal fluid biomarker examination are all adopted in AD diagnosis. Among the above methods, brain metabolic imaging and cerebrospinal fluid biomarker examination are both traumatic for human body, especially for advanced AD patients [5]. The recall rate of AD by EEG is influenced by onset age and dementia severity, and it shows some defects in the diagnosis of early AD [6]. PET can display the statuses of cerebrospinal fluid in the hippocampus and sulcus, but its definition and diagnostic capacity are poorer than those of MRI [7], which is the effective auxiliary method of the diagnosis of early AD [8].

The performance of machine learning algorithm is improved and enhanced by the constantly accumulated data to seek the optimal model. The algorithm is widely applied in data analysis and mining, mode recognition, bioinformatics, and medical treatment [9]. As the method that represents the technology level of integrated learning, random forest (RF) algorithm demonstrates unique advantages in processing high-dimension data. The results of the current studies show that RF can predict multiple diseases very accurately as a combined classifier, and it possesses high tolerance of abnormal values and noises. Besides, the overfitting of RF is rare [10]. RF consists of many decision trees (DT). Therefore, DT also shows potential values in the diagnosis of early AD [11]. In addition, some researchers point out that the classification abilities of MCI and AD by support vector machines (SVM) models are both excellent with the classification accuracy reaching as high as 82.0% [12]. However, current machine learning algorithm-based models are all adopted in AD diagnosis, while early AD prediction models are seldom studied. In addition, it is unknown which algorithm shows more advantages in early AD prediction.

To conclude, machine learning algorithm-based models showed significant advantages in AD diagnosis. However, there were few studies on the prediction of early AD by these models, and it was still unknown which algorithm demonstrated more advantages in early AD prediction. Hence, the MRI images of AD patients were included as the research objects. The AD prediction models of RF, DT, and SVM were established based on the analysis of hippocampal volume changes, and the application values of different models in early AD prediction were discussed to provide a referable basis for the diagnosis and treatment of AD patients.

## 2. Materials and Methods

### 2.1. Experimental Data and Grouping

American Alzheimer's disease neuroimaging initiative (ADNI) database was selected as the research objects. A total of 84 qualified research objects were selected randomly from serial numbers between 4801 and 5315. According to clinical dementia rating (CDR) [13] score and the diagnostic standards of *American Diagnostic and Statistical Manual of Mental Disorders* [14], all the patients were rolled into three groups, including cognitive function normal group (normal group), early mild cognitive impairment group (e-MCI group), and later mild cognitive impairment group (l-MCI group). Each group included 28 cases.

The inclusion standards of normal group were as follows: no memory loss; CDR scores were 0 points; barrier-free daily activities; normal cognitive function; and no dementia occurs.

The inclusion standards of e-MCI group were as follows: CDR scores were 0.5 points; no other cognitive disorders occur; daily activities were generally barrier-free; no dementia occurs; and delayed recall (DR) scores 20 minutes after logical memory test (LMT) were as follows. The cases educated for 16 years or longer were scored between 9 and 11 points. Those educated for 8 to 15 years were scored between 5 and 8 points. Those educated for 0 to 7 years were scored 3 or 4 points.

The inclusion standards of I-MCI group were similar to those of e-MCI group. Because cognitive function level was closely related to education level, LMT-DR scores were different. LMT-DR scores of I-MCI group were shown below. The cases educated for 16 years and longer were scored 8 points or less. Those educated for 8 to 15 years were scored 4 points or less. Those educated for 0 to 7 years were scored 2 points or less.

### 2.2. Experimental Data Preprocessing

Before the feature extraction and classification of MRI images, they needed to be preprocessed. The preprocessing of MRI images mainly included the following steps. The first step was the removal of skulls from MRI images by brain surface extractors. The second step was spatial standardization by FreeSurfer. The third step was the segmentation of axial MRI images into multiple subimages, the search for the maximum peak of subimage grayscale value histograms as the reference grayscale value of subimage white matters, and the smoothness processing of MRI images. The fourth step was the segmentation of brain tissues according to grayscale. The fifth step was the feature extraction according to segmentation results.

### 2.3. SVM Prediction Model Algorithm

SVM transformed the input space into a high-dimension space by nonlinear transformation and then obtained the optimal linear classification surface in the new space [15]. The given linear separable training set *A* was expressed by

(1) $$\begin{array}{c} A=\left\{\left(x_{i},y_{i}\right),i=1,2,\cdots l\right\},x_{i}\in R_{\text{n}},y_{i}\in \left\{-1,1\right\}. \end{array}$$

In equation (1), *x*_*i*_ referred to the *i*^th^ training sample, *y*_*i*_ represented the actual label of the *i*^th^ training sample, and *l* denoted the number of training samples.

SVM was aimed at searching for a decision function *f*(*x*) to separate training sets. The linear separable issue was expressed by classification hyperplane in

(2) $$\begin{array}{c} \left(\omega \cdot x\right)+b=0. \end{array}$$

In equation (2), *ω* denoted weight vectors and *b* referred to deviation items.

The core idea of SVM was the control of the promotion ability, and then, the classification interval maximization of classification hyperplane was transformed by

(3) $$\begin{array}{c} \min\frac{1}{2}{\left\|\omega \right\|}^{2} \end{array}$$

(4) $$\begin{array}{c} \text{s}.\text{t}:y_{i}\left[\left(\omega \cdot x_{i}\right)+b\right]\geq 1,\;i=1,2,\cdots l \end{array}$$

In equation (4), *x*_*i*_ referred to the input vector of the dimension *m* and *y*_*i*_ meant the label of samples.

As to approximate linear separable issues, the slack variable was introduced to transform the issues into the standard classification. A nonlinear mapping was introduced for linear inseparable issues, and low-dimension linear inseparable issues were transformed into high-dimension feature spatial linear separable issues. At last, the standard classification was adopted to obtain solutions. To avoid the complex calculation in high-dimension space, SVM adopted the kernel function *K*(*x*, *y*) to replace the inner product *Φ*(*x*)*Φ*(*y*) in the high-dimension space. Equation (5) was expressed as follows.

(5) $$\begin{array}{c} \min\left\{\frac{1}{2}{\left\|\omega \right\|}^{2}+\text{C}\overset{l}{\underset{i=1}{\sum }}\alpha_{i}\right\} \end{array}$$

(6) $$\begin{array}{c} \text{s}.\text{t}:y_{i}\left[\left(\omega \cdot x_{i}\right)+b\right]\geq 1‐\alpha_{i},\;i=1,2,\cdots l \end{array}$$

In equations (5) and (6), *C* represented the penalty coefficient adopted to balance classification intervals and misclassification specific gravity and *a*_*i*_ denoted slack variables.

Lagrange method was adopted to transform the above issues into a quadratic programming issue, and then the calculation method was expressed by

(7) $$\begin{array}{c} \min\frac{1}{2}\overset{l}{\underset{i=1}{\sum }}\overset{l}{\underset{i=1}{\sum }}\alpha_{i}\alpha_{j}y_{i}y_{j}K\left(x_{i}x_{j}\right)-\overset{l}{\underset{j=1}{\sum }}\alpha_{j} \end{array}$$

(8) $$\begin{array}{c} \text{s}.\text{t}.\overset{l}{\underset{i=1}{\sum }}y_{i}\alpha_{i}=0,0\leq \alpha_{i}\leq C,\;i=1,2,\cdots l \end{array}$$

The above two equations were solved, and then, equation (9) was obtained as follows.

(9) $$\begin{array}{c} f\left(x\right)=\mathrm{sgn}\left\{\overset{l}{\underset{i=1}{\sum }}\alpha_{i}y_{i}K\left(x_{i}\cdot x\right)+b\right\}. \end{array}$$

Based on functional theory, the kernel function corresponded to the inner product in a certain transformation space if it met Mercer conditions. Then, the classification function of SVM was expressed by

(10) $$\begin{array}{c} f\left(x\right)=\mathrm{sgn}\left\{\overset{k}{\underset{i=1}{\sum }}\alpha_{i}^{*}y_{i}K\left(x_{i}\cdot x\right)+b^{*}\right\}. \end{array}$$

In equation (10), *α*_*i*_^∗^ referred to Lagrange multipliers and *b*∗ represented classification thresholds.

In the research, the radial basis function was selected as the kernel function. As equation (11) indicated, *γ* referred to Gaussian kernel parameters.

(11) $$\begin{array}{c} K\left(x,x_{i}\right)=\exp\left(-\gamma {\left\|x-x_{i}\right\|}^{2}\right). \end{array}$$

If a group of training samples could be separated by an optimal classification surface, the expected classification error rate of test samples met the following conditions, which were shown in

(12) $$\begin{array}{c} E\left[P\left(\text{error}\right)\right]\leq \frac{E\left(\text{SV}\right)}{n}. \end{array}$$

In equation (12), *n* referred to the number of training sets, SV denoted support vectors, *E*[*P*(error)] represented the expectation of the classification error rate of test samples, and *E*(SV) stood for the expectation of the number of SV. The accuracy discriminant weight *w*_*t*_ was expressed by

(13) $$\begin{array}{c} w_{t}=1-\frac{E\left(SV\right)}{n}。K\left(x,x_{i}\right)=\phi \left(x\right)\phi \left(x_{i}\right). \end{array}$$

### 2.4. DT and RF Prediction Model Algorithms

DT classified data based on the tree structure. Data was divided into different regions based on distribution features. Measurement purity was commonly adopted to show classification effects, and the common standard of measurement purity was information entropy [16], whose calculation method was demonstrated by

(14) $$\begin{array}{c} E=-p*\log\left(p\right)-\left(1-p\right)*\log\left(1-p\right). \end{array}$$

In equation (14), *p* denoted the true sample proportion in current nodes. It was assumed that the reliability of the result *p*_*i*_ of the *i*^th^ sample was expressed by

(15) $$\begin{array}{c} L_{\text{i}}={p^{i}}^{y_{i}}*{\left(1-p_{i}\right)}^{1-y_{i}}y_{i}. \end{array}$$

In equation (15), *y*_*i*_ referred to the class label of the *i*^th^ sample. It was assumed that the probability of accurate classification followed Bernoulli distribution, and then, the target function of data sets was expressed by

(16) $$\begin{array}{c} T=\overset{l}{\underset{\text{i}=1}{∐}}\left[{p^{i}}^{y_{i}}*{\left(1-p_{i}\right)}^{1-y_{i}}y_{i}\right]. \end{array}$$

The logarithm and inverse of the above equation were obtained, and then, the calculation method of the target function of data sets was transformed as

(17) $$\begin{array}{c} f=-\log\left(T\right). \end{array}$$

The minimization solution of the function was the same thing as the maximization solution of the original function, and then, the issue was transformed into the function parameter of extremum solution, whose expression was shown in

(18) $$\begin{array}{c} p_{k}=\frac{\sum_{i=1}^{m}y_{i}}{m}. \end{array}$$

In equation (18), *m* denoted all samples of this node and *p*_*k*_ referred to the proportion of true samples. The target function of data sets was transformed into

(19) $$\begin{array}{c} f_{k}=\overset{m}{\underset{i=1}{\sum }}y_{i}\log p_{k}-\overset{m}{\underset{i=1}{\sum }}\left(1-y_{i}\right)\log\left(1-p_{k}\right). \end{array}$$

The normalization of node samples was adopted to eliminate the influences of sample points on the number of samples [17], and then, the calculation method of the target function of data sets was expressed by

(20) $$\begin{array}{c} \frac{f_{k}}{m}=p_{k}\log p_{k}-\left(1-p_{k}\right)\log\left(1-p_{k}\right). \end{array}$$

RF was a combined classifier algorithm synthesized by many DT classification models. RF added the differences among classification models by constructing different training sets to improve the prediction effects of classification models [18]. The classification decision of the models was expressed by

(21) $$\begin{array}{c} R\left(x\right)=\arg_{\varepsilon }^{\max}\overset{k}{\underset{i=1}{\sum }}A\left[r_{i}\left(x\right)=Y\right]. \end{array}$$

In equation (21), *R*(*x*) referred to combined classification models, *k* represented the number of training, *r*_*i*_ denoted a DT classification model, and *Y* stood for target variables.

### 2.5. Establishment of Machine Learning Prediction Models

In the research, the implementation of machine learning algorithm model transformation and data prediction was based both on Matlab2016a platform. Data preprocessed by MRI was imported, and MRI data were normalized. After that, 20 groups of test and training sets were selected, respectively, for the training and classification test on data, which was aimed at establishing prediction models. Besides, the prediction accuracy, sensitivity, and specificity parameters of prediction models were calculated under test sets.  Figure 1 demonstrated the specific process of early AD prediction based on machine learning algorithms as follows.

### 2.6. Observation Indexes

The volumes of hippocampal subregions, including left CA1, left CA2-3, left CA4-DG, left presubiculum, left tail, right CA2-3, right CA4-DG, right presubiculum, and right tail in different groups, were compared. The correlation between different hippocampal volumes and LMT-DR was analyzed. The predictive accuracy of early AD by prediction models established based on different algorithms and the predictive accuracy of different MRI feature indexes were analyzed. Besides, the predictive accuracy, sensitivity, and specificity of early AD by different models were compared.

### 2.7. Statistical Methods

After being preprocessed by MRI image data, a total of 16 volume indexes in hippocampal subregions were obtained. All data were analyzed by statistical product and service solutions (SPSS) software. In addition, a one-way variance analysis was performed on the data complying with normality and homoscedasticity. The least significant difference (LSD) method was adopted in the comparison among groups. In contrast, the data that did not conform to normality and homoscedasticity test was processed by Kruskal-Wallis *H* nonparametric test. Pairwise comparisons among multiple independent samples were tested by Nemenyi method. Besides, MRI feature data with significant differences among groups were processed by multiple linear regression analysis. *α* = 0.05 was set as the test level, and *P* < 0.05 indicated that the differences showed statistical meaning.

## 3. Results

### 3.1. Analysis of Results of MRI Data Preprocessing

After MRI data preprocessing and feature extraction, a total of 16 volume indexes in hippocampal subregions. After the multiple comparisons by a one-way variance analysis and LSD method, pairwise comparisons among groups demonstrated that 8 volume indexes in hippocampal subregions showed differences. The volumes of hippocampi in e-MCI group, including left CA1, left CA2-3, left CA4-DG, left presubiculum, left tail, right CA2-3, right CA4-DG, right presubiculum, and right tail, were all smaller than those in normal group, and the comparison between two groups demonstrated significant differences (*P* < 0.01). The volumes of hippocampi in I-MCI group, including left CA1, left CA2-3, left CA4-DG, left presubiculum, left tail, right CA2-3, right CA4-DG, right presubiculum, and right tail, were all decreased compared with those in e-MCI group, and the comparison between two groups revealed obvious differences (*P* < 0.01). Besides, the corresponding volumes of hippocampi in hippocampal subregions in I-MCI group were significantly reduced compared with those in normal group, and the comparison between the two groups indicated extremely significant differences (*P* < 0.01). All the results of the above comparisons were illustrated in Figure 2.

### 3.2. Relevance Analysis of Volume Changes in Hippocampal Subregions and LMT-DR

The relevance between hippocampal volumes and LMT-DR in behavioristics was analyzed. In left hippocampal subregions, the volumes of 3 subregions, including left CA1, left CA2-3, and left CA4-DG, were all correlated with LMT-DR scores, which were shown in Figures 3, 4, and 5. The volumes of left CA1 regions were positively correlated with LMT-DR scores significantly (*R*^2^ = 0.1702, *P* < 0.001), the volumes of left CA2-3 regions were positively correlated with LMT-DR scores significantly (*R*^2^ = 0.3779, *P* < 0.001), and the volumes of left CA4-DG regions were positively correlated with LMT-DR scores significantly (*R*^2^ = 0.1607, *P* < 0.001).

The volumes of 3 subregions in right hippocampal subregions, including right CA2-3, right CA4-DG, and right presubiculum, were all correlated with LMT-DR scores, which were demonstrated in Figures 6, 7, and 8. The volumes of right CA2-3 regions were positively correlated with LMT-DR scores significantly (*R*^2^ = 0.1620, *P* < 0.001), the volumes of right CA4-DG regions were positively correlated with LMT-DR scores significantly (*R*^2^ = 0.0426, *P* < 0.001), and the volumes of right presubiculum regions were positively correlated with LMT-DR scores significantly (*R*^2^ = 0.1309, *P* < 0.001).

### 3.3. Analysis of AD Prediction Results by Different Models

Different models established in the research were adopted to analyze the prediction results of normal, e-MCI, and l-MCI groups, respectively. The numbers including 0, 1, and 2 were adopted to symbolize normal, e-MCI, and I-MCI groups, respectively.  Figure 9 displayed the prediction of different types of results by DT models. The prediction results of 8 data were inconsistent with the actual results, and the prediction accuracy of training set samples reached 86.67%.

Figure 10 presented the prediction of different types of results by SVM models. The prediction results of 4 data were inconsistent with the actual results, and the prediction accuracy of training set samples amounted to 93.33%.

Figure 11 demonstrated the prediction of different types of results by RF models. The prediction result of 1 data was inconsistent with the actual result, and the prediction accuracy of training set samples amounted to 98.33%.

### 3.4. Comparison of Prediction Accuracy of Different MRI Feature Indexes

The e-MCI and l-MCI were predicted by RF, SVM, and DT models based on the volume change parameters of different hippocampal subregions, and the prediction results were compared and analyzed (Figure 12). In the prediction of the volume changes in different hippocampal subregions, the prediction accuracy by RF models was higher than that by SVM and DT models. Based on left CA1 and left CA2-3 volume changes, the prediction accuracy of e-MCI by RF models was higher than that by DT models (*P* < 0.05). Besides, the prediction accuracy of e-MCI based on left CA4-DG, right CA2-3, and right CA4-DG volume changes by RF models was significantly higher than that by DT models (*P* < 0.01). Based on left CA2-3 volume changes, the prediction accuracy of l-MCI by RF models was higher than that by DT models (*P* < 0.05), and the prediction accuracy of l-MCI was obviously higher than that by DT models, which was based on left CA4-DG, right CA2-3, and right CA4-DG volume changes (*P* < 0.01). What is more, it was observed that the prediction accuracy of e-MCI and l-MCI by different models based on left CA4-DG, right CA2-3, and right CA4-DG volume changes was remarkably higher than that by right presubiculum, and the comparison between two values showed significant differences (*P* < 0.01).

### 3.5. Comparison of Prediction Performances of Different Machine Learning Algorithms

RF, SVM, and DT models were adopted to predict e-MCI, as shown in Figure 13. The predictive accuracy of e-MCI by RF, SVM, and DT models reached 95.68%, 82.58%, and 78.25%, respectively. The predictive sensitivity of e-MCI by the three models amounted to 88.16%, 68.34%, and 68.52%. The predictive specificity of e-MCI by the three algorithms was 93.05%, 79.81%, and 81.57%. The predictive accuracy, sensitivity, and specificity of e-MCI by RF model were all obviously higher than those by DT model (*P* < 0.01). Besides, the comparison of the predictive accuracy, sensitivity, and specificity of e-MCI by DT model and by SVM model showed no statistical differences (*P* > 0.05).

## 4. Discussion

Early AD patients might suffer from memory impairment, depression, sleep arousal disorders, and sexual dysfunction [19, 20]. With MCI developing into AD, the decrease in hippocampal volumes was aggravated [21]. In the research, early AD prediction models were established based on multiple machine learning algorithms, and the prediction performances of different models were compared to seek the optimal prediction model. As an essential data preprocessing step, feature selection can solve dimension disaster issues in real tasks [22]. In the research, MRI image data was preprocessed, and its features were extracted to obtain 16 volume indexes in hippocampal subregions. After multiple comparisons, by one-way variance analysis and LSD method, pairwise comparisons among groups demonstrated that a total of 8 volume change indexes in hippocampal subregions showed differences. The results of the research showed that the volumes of hippocampi in e-MCI group, including left CA1, left CA2-3, left CA4-DG, left presubiculum, left tail, right CA2-3, right CA4-DG, right presubiculum, and right tail, were all smaller than those in normal group (*P* < 0.01). The volumes of hippocampal subregions corresponding to hippocampi in I-MCI group were all decreased compared with those in e-MCI group (*P* < 0.01). Besides, the corresponding volumes of hippocampal subregions in I-MCI group were significantly reduced compared with those in normal group (*P* < 0.001). The above results demonstrated that the severity of AD disease was positively correlated with the volume changes in hippocampal subregions. In addition, the further analysis of the relevance between hippocampal volumes and LMT-DR in behavioristics revealed that the volumes of subregions, including left CA, left CA2-3, left CA4-DG, right CA2-3, right CA4-DG, and right presubiculum, were all positively correlated with LMT-DR scores significantly. The results showed that the volume reduction in gray matters in CA2-3 and CA4-DG hippocampal subregions could be viewed as the potential indexes of evaluating patient memory impairment. According to some studies, the hippocampal subregions including CA2-3, CA4-DG, and subiculum also could be used to reflect or predict disease progress [23]. Besides, these hippocampal subregions might be more suitable for predicting AD [24]. There were some similarities between the research result and these findings. The left and right CA2-3 and CA4-DG subregions were both related to the development of AD. In addition, it was found out that the region of right presubiculum was also correlated with the impairment of memory function based on deep learning model. The region could be used as a potential AD prediction index.

In the training of data sets, RF could introduce two randomness to avoid overfitting [25]. Besides, it showed advantages in antinoise performance [26]. RF could process continuous and discrete data simultaneously [27] and possess significant advantages in processing high-dimension data, such as simplicity, realizability, and low computing cost [28]. The results of the research revealed that the prediction accuracy of RF training set samples reached 98.33%. Furthermore, the prediction accuracy of e-MCI based on left CA4-DG, right CA2-3, and right CA4-DG volume changes was obviously higher than that by DT models (*P* < 0.01). The prediction accuracy, sensitivity, and specificity of e-MCI by RF models were all remarkably higher than those by DT models (*P* < 0.01). The above results demonstrated that RF showed excellent performance in predicting the risk transformation from e-MCI to I-MCI.

## 5. Conclusion

Based on machine learning method, early AD was predicted by hippocampal subregion volume changes. The result indicated that RF model showed high predictive performance in predicting the risk of transformation from e-MCI to l-MCI among different machine learning methods. However, there were still some advantages in this research. For example, the research was implemented based only on ADNI public database without further clinical verification of RF performance. In future research, more early AD cases needed to be included, and early AD should be predicted by RF models to verify its correctness. To conclude, effective early AD prediction models were established by hippocampal subregion volume changes, which was based on RF. The establishment of early AD prediction model provided certain references for the diagnosis and treatment of AD patients.

## Figures and Tables

**Figure 1:** Machine learning model-based early AD prediction process.

**Figure 2:** Comparison of hippocampal volumes in different groups by MRI data. (a) demonstrated the comparison of left tail hippocampal subregion volumes in different groups, and (b) showed the comparison of right tail hippocampal subregion volumes in different groups. ∗ indicated that the comparison with normal group showed significant differences, *P* < 0.01; ∗∗ meant that the comparison with normal group demonstrated extremely significant differences, *P* < 0.001; # showed that the comparison with e-MCI group revealed significant differences, *P* < 0.01.

**Figure 3:** Relevance analysis of left CA1 region volumes and LMT-DR scores.

**Figure 4:** Relevance analysis of left CA2-3 region volumes and LMT-DR scores.

**Figure 5:** Relevance analysis of left CA4-DG region volumes and LMT-DR scores.

**Figure 6:** Relevance analysis of right CA2-3 region volumes and LMT-DR scores.

**Figure 7:** Relevance analysis of right CA4-DG region volumes and LMT-DR scores.

**Figure 8:** Relevance analysis of right presubiculum region volumes and LMT-DR scores.

**Figure 9:** Analysis of prediction results by DT models.

**Figure 10:** Analysis of prediction results by SVM models.

**Figure 11:** Analysis of prediction results by RF models.

**Figure 12:** Comparison of prediction accuracy by different algorithms. (a) showed the comparison of the prediction accuracy of e-MCI by different models based on different hippocampal subregions volume changes, and (b) demonstrated the comparison of the prediction accuracy of I-MCI by different models based on different hippocampal subregions volume changes. ∗ indicated that the comparison with DT models showed statistical differences, *P* < 0.05; ∗∗ showed that the comparison with DT models revealed significant differences, *P* < 0.01; ∗∗∗ suggested that the comparison with DT model demonstrated extremely significant differences, *P* < 0.001.

**Figure 13:** Comparison of prediction performances of different machine learning algorithms. ∗∗ indicated that the comparison with DT models showed significant differences, *P* < 0.01.

## Data Availability

The data used to support the findings of this study are available from the corresponding author upon request.
